The article "Multimodal Neuroelectrophysiological Monitoring Combined with Robot-Assisted Placement of a Transiliac–Transsacral Screw for the Treatment of Transforaminal Sacral Fractures" was published in 2022. Journal: Biomed Res Int.

# Multimodal Neuroelectrophysiological Monitoring Combined with Robot-Assisted Placement of a Transiliac–Transsacral Screw for the Treatment of Transforaminal Sacral Fractures

**DOI:** 10.1155/2022/3383665

**Published:** 2022-07-23

**Authors:** Pengfei Wang, Kun Yang, Huaguang Qi, Xinan Yan, Chen Fei, Xuemei Liu, Xing Wei, Hu Wang, Yahui Fu, Hongli Deng, Kun Zhang, Yan Zhuang

**Affiliations:** ^1^Department of Orthopedics and Traumatology, Xi'an Honghui Hospital, Xi'an JiaoTong University Health Science Center, Xi'an, China; ^2^Department of Hand and Foot Microsurgery, The First Hospital of Yulin, Yulin, China; ^3^Department of Functional Examination, Xi'an Honghui Hospital, Xi'an JiaoTong University Health Science Center, No. 555, East Friendship Road, Xi'an City, Shaanxi Province, China

## Abstract

**Objective:**

This study aimed to evaluate the safety and efficacy of the fixation of transforaminal sacral fractures using TiRobot-assisted transiliac-transsacral (TITS) screws under multimodal neuroelectrophysiological monitoring (MNM).

**Methods:**

From January 2019 to May 2021, 22 patients (17 male and 5 female patients) with transforaminal sacral fractures who were treated with closed reduction and placement of TiRobot-assisted TITS screws under MNM were retrospectively evaluated. The average age of the patients was 43.32 ± 11.40 years (range: 19–63). The patients received MNM, including somatosensory-evoked potentials (SEPs), motor-evoked potentials (MEPs), and electromyographic monitoring (EMG), prior to surgery, during closed reduction and the placement of the guidewire and TITS screw, and at the end of surgery. The operation was adjusted according to the MNM results.

**Results:**

Overall, 22 TITS screws were inserted in 22 patients, including 5 TITS screws in the S1 body and 17 TITS screws in the S2 body. The average time needed for screw placement was 27.95 ± 6.84 mins, and the average frequency of X-ray fluoroscopy exposures was 31.00 ± 5.56 for each patient. Anterior ring fixation was performed in 4 patients using an external fixator, in 5 patients using cannulated screws, and in 13 patients using reconstruction plates. The mean follow-up time was 14.46 ± 2.46 months (12–20 months). Tornetta and Matta radiographic outcomes were excellent in 10 patients, good in 9 patients, fair in 2 patients, and poor in 1 patient. The proportion of excellent and good ratings was 86.36%. At the final follow-up, the average Majeed score was 82.18 ± 14.52, with clinical outcomes that were excellent in 9 patients, good in 9 patients, fair in 1 patient, and poor in 3 patients. The proportion of excellent and good ratings was 82.82%. Preoperatively, the amplitude of the SEP on the injured side was lower than that on the contralateral side before reduction in 9 patients (>50%). In this study, no screw was mistakenly inserted into the sacral canal, and no surgical site infection occurred.

**Conclusion:**

MNM combined with TiRobot assistance can safely implant TITS screws and can effectively identify the neurological function of patients under anesthesia and reduce iatrogenic nerve injury.

## 1. Introduction

Due to the aging of the population, the yearly incidence rate of pelvic fractures increased from 58 per 100,000 person-years in 2001 to 73 per 100,000 person-years in 2016 [1]. The incidence of unstable pelvic fracture is approximately 17–30% and is often associated with nerve injury [2, 3]. In patients with unstable pelvic ring or nerve injury, open reduction and internal fixation (ORIF) has been used to reduce the time in bed, relieve neurological symptoms, and reduce the disability rate [4, 5]. However, ORIF is often associated with greater trauma, more extensive soft tissue dissection, more blood loss, and a high risk of surgical site infection [6–8]. Therefore, the use of minimally invasive treatment methods for pelvic fractures, such as sacroiliac screws, is widely supported by scholars [9–11]. However, sacroiliac screws have a high failure rate in the fixation of posterior pelvic ring fractures [12, 13]. A previous finite element analysis reported that lengthening sacroiliac screws can improve the fixation strength of the posterior pelvic ring [14]. However, percutaneous placement of TITS screws through closed reduction is highly technically demanding and involves longer operation times, multiple fluoroscopy exposures, and risk of sacral nerve injury [15].

Recently, with the development of computer-assisted orthopedic surgery (CAOS), orthopedic robots have been widely applied in trauma and orthopedic surgery and have obvious advantages in accurate sacroiliac screw placement [16]. However, it remains unknown whether sacral nerve injury occurs during fracture reduction, guidewire insertion, or screw placement after the patient was placed under general anesthesia. MNM has been fully developed during spinal surgery because it provides real-time monitoring information of nerve function and timely detection of nerve injury for surgeons. Therefore, MNM ensures the safety of surgery, which has been favored by an increasing number of orthopedic surgeons [17, 18]. The goal of intraoperative neuroelectrophysiological monitoring is to identify early changes in neural activity to guide procedural actions and adjustments that ultimately may prevent definitive injury to nerves. However, neurophysiologic monitoring has not enjoyed the same widespread acceptance among trauma surgeons as among spine surgeons. A survey of trauma surgeons demonstrated that only 15% use monomodal neuroelectrophysiological monitoring [19]. Although MNM has been reported to be safe and effective in predicting iatrogenic sciatic nerve injury during acetabular and pelvic fracture fixation, its application to pelvic fracture fixation has been limited [18].

In the current study, we hypothesized that MNM combined with TiRobot assistance can lead to the safe implantation of TITS screws and can timely and effectively identify changes in patients under anesthesia.

## 2. Patients and Methods

This study was approved by the appropriate Institutional Review Board. All patients signed informed consent forms. All patients who were admitted to our institution and fulfilled the following criteria were enrolled in the study. The inclusion criteria were as follows: (1) adult patients aged ≥18 years with unstable pelvic fractures; (2) unstable pelvic fractures combined with transforaminal sacral fractures; (3) sacral fractures were fixed using TITS screw(s) with the TiRobot assistant; (4) neuroelectrophysiological monitoring was performed; and (5) complete follow-up was available. Patients with an associated acetabular fracture were excluded.

Preoperatively, the patients underwent routine AP view, inlet and outlet views, computerized tomography (CT) scan, and 3D reconstruction of the pelvis to assess the fracture pattern according to the AO/OTA classification. Preoperative 3D CT was used to evaluate the presence of a dysmorphic sacrum. Coronal and axial CT scans were used to evaluate the size of the corridors.

Low molecular weight heparin (LMWH) was prescribed as chemoprophylaxis for deep vein thrombosis during the perioperative period. Antibiotics were administered 30 min preoperatively to prevent infection.

### 2.1. Surgical Technique

All operations were performed by the same surgeons (PFW and YZ). Patients were placed in the supine position on a radiolucent table after successful induction of anesthesia. Anesthetic agents and administration methods that have less impact on muscle relaxants were used. Electrodes were placed at the monitoring site. The device (Cascade Elite, Cadwell Industries, Inc., USA) was connected, and the electrophysiological monitoring program was started. TiRobot (Beijing Tinavi Medical Technologies Co., Ltd. China) was connected, and the patient's information was registered on a computer. The sacral fractures were reduced by closed manipulation. Acceptable reduction was radiographically confirmed and was maintained by traction, external fixators or a Starr frame until the screw application was complete. The tracer was firmly fixed to the anterior superior iliac spine of the contralateral side. The mechanical arm with a sterile protective sleeve was moved and fixed to the injured side. The mechanical arm tracer was placed on the patient's surgical site for subsequent fluoroscopy. Intraoperative fluoroscopy images containing the robot positioning markers were obtained and transmitted to the computer. The placement of TITS screws was planned on the computer. Under the control of the computer, the mechanical arm with the guide sleeve was moved to the operation site. A small incision (approximately 1 cm in length) was made, and the subcutaneous and muscular tissues were bluntly separated. The tip of the sleeve was pressed to the bone cortex, and a 2.5 mm ×400 mm Kirschner wire was inserted as the guidewire. The satisfactory positioning of the guidewire was confirmed using radiography. An extended 7.3-mm cannulated screw (IRENE Medical Instrument Co., Ltd., Tianjin, China) was inserted. The position of the screw was confirmed using fluoroscopy, the guidewire was removed, and the incision was sutured. During the operation, the electrophysiologist supervised the entire process.

### 2.2. Intraoperative Electrophysiological Monitoring

The international 10/20 system was used for the SEP recording electrode [20]. The lower extremity SEP recording electrode was located at the Cz′point (an improved area 2 cm behind the Cz point). The reference electrode was placed at the Fz point, and the interelectrode impedance was <5 k*Ω*. The stimulation electrodes were located in the area innervated by the posterior tibial nerve. The parameter settings were as follows: constant current pulse stimulation, 20–40 mA stimulation intensity, 0.1–0.2 ms stimulation duration, 3.1 Hz stimulation frequency, average of 200 signal stacking times, and filtering at 30 Hz–3 KHz.

Transcranial electrical stimulation was used for MEP monitoring. Stimulating electrodes were placed on the C1 and C2 points (the scalp area corresponding to the motor cortex related to lower extremities) and mutually referenced. The recording electrodes were placed in the pretibial muscle, extensor hallucis longus, gastrocnemius muscle, hallucis adductor, and anal sphincter. Myogenic MEPs were obtained from muscle recordings after transcranial electrical stimulation. The TOF value was measured, the stimulation intensity was increased from small to large, and the stable MEP was subject to a maximum of 400 V. The stimulation method was multipulse square wave stimulation, with 5–8 stimulation strings and 1–6 ms pulse intervals.

EMG monitoring records the spontaneous EMG activity generated when nerve-innervated muscles are stimulated. With pass-through filtering at 10–1000 Hz, nerve roots of L5, S1, and S2 were selected as they innervate the tibialis anterior muscle, great extensor muscle, gastrocnemius muscle, and anal sphincter, and recording electrodes were placed for continuous intraoperative monitoring.

Regarding the criteria and treatment of nerve injury during monitoring [21], neuroelectrophysiological examination (including SEP, MEP, and EMG) was performed preoperatively to determine whether there was nerve injury and the extent of injury. The baseline setting was thus established. Continuous multimodal electrophysiological monitoring was carried out during the operation, with a focus on closed reduction, guidewire placement, drilling, and screw placement. The electrophysiologist closely monitored whether sacral nerve injury or injury aggravation occurred. The following signals were examined during electrophysiological monitoring and considered nerve injury: (1) abnormal explosive EMG related to the surgical operation; (2) MEP monitoring, which adopted an “all or none” judgment standard, with a stimulus threshold >100 V higher than the baseline threshold; and (3) SEP amplitude reduced by 50% or the incubation period prolonged by 10%. The false positives caused by other nonsurgical factors were excluded and analyzed, and any possible injury caused by the operation was remedied and repaired as soon as possible. At the end of the operation, the neuroelectrophysiological monitoring results were observed again, and the operation was completed when no abnormalities were found.

### 2.3. Postoperative Management

Prophylactic use of antibiotics was continued for 48–72 hours postoperatively. Low-molecular-weight heparin (LMWH, 4100 U, once daily, GlaxoSmithKline Co., UK) was routinely used for venous thromboembolism (VTE) prophylaxis during hospitalization, except for patients who had contraindications. At discharge from the hospital, the patients were prescribed 10 mg rivaroxaban once daily for 5 weeks postoperatively to prevent VTE. For VTE treatment, the dose of LMWH or rivaroxaban was adjusted according to the patient's body weight. The patients were given instructions about postoperative rehabilitation before discharge that included protected toe-touch weight-bearing activity for six weeks. After 6-8 weeks and a follow-up visit to the clinic, the patients were encouraged to gradually increase weight-bearing (Figures 1(a)–1(i)).

### 2.4. Data Collection

The following data were collected: (1) demographics: sex, age, and mechanism of injury; (2) fracture pattern: classified by AO/OTA classification; (3) Injury Severity Score (ISS); (4) associated injuries; (5) surgery-related variables: anterior ring fixation, operative time, estimated blood loss, and quality of the reduction (Tornetta and Matta's radiologic criteria); (6) final functional outcomes (Majeed score) [22]; and (7) complications: nerve injury, infection. The follow-up evaluations occurred at postoperative clinical visits after two weeks, four weeks, six weeks, eight weeks, three months, six months, one year, and annually thereafter.

The radiographic and functional outcomes were evaluated by an orthopedic traumatologist (XW) who was not involved in the care of the patients. This independent observer (XW) assessed reduction quality according to Tornetta and Matta criteria using the measurements of the displacement asymmetry, deformity index, vertical displacement, horizontal displacement, and diastasis of the pubic symphysis on radiographs and CT scans [23, 24]. The reduction was excellent when the residual displacement was 0–4 mm, good at 4–10 mm, fair at 10–20 mm, and poor at>20 mm. Clinical outcomes were evaluated using Majeed scores [22]. The scores were categorized as excellent (>85 points), good (70–84 points), fair (55–69 points), or poor (<55 points).

### 2.5. Statistics

The Statistical Package for Social Sciences (SPSS) software version 19.0 (IBM, Chicago, IL, USA) was used. Continuous variable data are presented as the means and standard deviations. Comparisons between preoperative neurological injury and final follow-up neurological injury were performed using the Wilcoxon signed-rank test.

## 3. Results

A total of 22 TITS screws were inserted in 22 patients, including screws in S1 in 5 patients and in S2 in 17 patients. The average time to place each screw was 27.95 ± 6.84 mins, and the frequency of fluoroscopy exposures per patient was 31.00 ± 5.56. Regarding the anterior ring fixation methods, external fixator fixation was performed in 4 patients, pubic ramus cannulated screw fixation was performed in 5 patients, and plate fixation was performed in 13 patients.

All patients were followed up, and the average follow-up time was 14.46 ± 2.46 months (12–20 months). Tornetta and Matta radiographic outcomes were excellent in 10 patients, good in 9 patients, fair in 2 patients, and poor in 1 patient. The proportion of excellent and good ratings was 86.36%. At the final follow-up, the average Majeed score was 82.18 ± 14.52, with clinical outcomes that were excellent in 9 patients, good in 9 patients, fair in 1 patient, and poor in 3 patients. The proportion of excellent and good ratings was 81.82%. The amplitude of the SEP potential on the affected side was lower than that on the opposite side before reduction in nine patients. There was no significant change in the amplitude of the wave after the operation compared to before reduction. In 4 patients, the amplitude of the SEP wave decreased during continuous heavy weight skeletal traction and maneuvers. One patient had a spontaneous burst of EMG activity when the guidewire was inserted. The other patients showed no significant changes in the SEP, MEP, or EMG amplitudes before, during, or after surgery. No screw penetrated into the sacral foramen or sacral canal. No surgical site infections were observed (Tables 1–3).

## 4. Discussion

The use of sacroiliac screws for minimally invasive treatment of sacral fractures and sacroiliac dislocation was first reported by Matta JM et al. [25]. Biomechanical studies have shown that sacroiliac screws have the biological properties of central fixation and stability, can resist vertical shear force and torsion, and are a feasible method for the treatment of unstable posterior pelvic ring injuries that have the advantages of less trauma, quick recovery, and satisfactory efficacy [25]. It is generally believed that the longer the sacroiliac screw length is, the better the load can be dispersed, the stress on the screw can be reduced, and the displacement can be resisted, which makes this an excellent choice for the treatment of transforaminal sacral fracture [26]. Extended sacroiliac screw fixation can effectively reduce the failure rate of internal fixation for Tile C fractures with poor stability [14, 27], let alone full-length TITS screw fixation. The TITS screw is a single screw that is used to fix a sacral fracture through the bilateral iliac crest, bilateral sacroiliac joints, and sacral body. Some authors have found that TITS screw fixation with bilateral iliac bones has a high control force [28]. However, the TITS screw must pass through the bilateral sacral wing area. Due to the narrow corridor, screw misplacement is more likely to occur with an increase in screw length, resulting in an increased possibility of iatrogenic injury of peripheral vascular nerves [15, 29]. In addition, during the placement of TITS screws, repeated fluoroscopy is required to ensure the safety of screw placement, which increases the radiation exposure to the medical staff and patients. Meanwhile, the accuracy of TITS screw placement is affected by factors such as inadequate fluoroscopic experience, trajectory deviation, and poor freehand stability. Therefore, to improve the accuracy and safety of TITS screw placement and to reduce the difficulty of the operation, we implanted TITS screws with the assistance of TiRobot. In this study, 22 TITS screws were inserted. The average placement time for each screw was 27.95 ± 6.84 mins. Wu et al. [30] reported that the average time spent on each screw was 60.3 ± 5.8 mins with freehand sacroiliac screw placement, which was much longer than the time spent in the current study. In the current study, although the average number of X-ray fluoroscopy exposures per patient was 31.00 ± 5.56, which was more than that in their study, the reduction procedure was included in the current study. Long T et al. [31] compared the efficacy of robot assistance with freehand sacroiliac screw placement and found that robot-assisted screw placement had the advantages of less trauma, less bleeding, and shorter operation time, which was similar to the findings in the current study. According to the Tornetta and Matta radiographic grades, the outcomes were excellent in 10 patients, were good in 9 cases, were fair in 2 cases, and were poor in 1 case. The proportion of excellent and good ratings was 86.36%, which was similar to a previous study [31]. At final follow-up, all patients recovered from neurological injury except for three severely injured patients. There were no instances of a screw penetrating the sacral foramen, sacral canal, or bone cortex. No surgical site infection was observed.

Transforaminal sacral fractures are prone to nerve injury [32], which occurs in as many as 29–60% of fracture cases [33]. In the current study, 40.9% (9/22) of patients presented with nerve injury preoperatively. With indirect reduction and percutaneous TITS screw fixation, finally, the neurological function showed significant recovery (Table 3). Reilly et al. [34] suggested that if a pelvic posterior ring fracture was displaced >10 mm, the risk of nerve and blood vessel injury during sacroiliac screw placement would be significantly increased. Similarly, there is a risk of sacral plexus injury during intraoperative reduction, traction, or insertion of sacroiliac screws. Furthermore, determining whether iatrogenic nerve injury occurs during surgery is difficult for surgeons, especially when the patients are under anesthesia. Intraoperative multimodal neuroelectrophysiological monitoring technology has been well developed in neurosurgery and spine surgery, which can provide real-time monitoring of nerve function for surgeons and timely detection of nerve injury, ensuring surgical safety. Thus, monitoring is currently favored by an increasing number of orthopedic surgeons [17, 35–38]. Nevertheless, few studies have reported neuroelectrophysiological monitoring during pelvic surgery [18, 39]. SEP and MEP signals during surgery are affected by many factors, including the dose and type of anesthetic drugs. To obtain high-quality SEP and MEP signals, sudden administration of large doses of drugs or changes of medication type should be avoided during surgery after communication with an anesthesiologist, and an intravenous pump should be used to maintain a constant dose administration. When electrophysiological monitoring provided an alert, the operation was immediately stopped, changes in SEP, MEP, and EMG waveforms were observed, and the operation was continued after the possibility of nerves being stretched or compressed was excluded. The results showed that the SEP amplitude on the injured side decreased to baseline in 4 patients during heavy weight traction and maneuvers and gradually recovered after relaxation and revised maneuvers. One patient had a spontaneous burst of EMG activity when the guidewire was inserted. The guidewire was redirected, and EMG activity recovered. The other patients had no abnormal changes in SEP, MEP, or EMG during the entire operation, which suggested that there was no iatrogenic nerve injury or further aggravation of nerve injury during the operation. Hence, we recommend routine multimodal neuromonitoring for the placement of TITS screws in the treatment of transforaminal sacral fractures and suggest the use of the multimodal neuromonitoring described in this study to monitor the sensory and motor pathways if neuromonitoring is chosen. Multimodal neuroelectrophysiological monitoring can maximize the reliability of identifying neural injury and preventing iatrogenic nerve injury, thus improving the safety and effectiveness of surgery.

### 4.1. Limitations

This study has several limitations. First, it was a retrospective study, making it susceptible to examiner bias. Second, one of the more limiting factors of a retrospective chart review relates to dependence on postoperative motor examination results as performed by independent pelvic surgeons who were not involved in the treatment with specific assessment criteria. Third, we report on a relatively short follow-up and small sample of 22 pelvic injuries that may be too small to determine if it would be possible to reliably identify a nerve injury. Fourth, there was no control group to which the merits in the current study could be compared.

## 5. Conclusion

Robot-assisted TITS screw placement in the treatment of transforaminal sacral fractures is accurate and minimally invasive, with fewer fluoroscopy exposures and reduced radiation exposure. Intraoperative neuroelectrophysiological monitoring is a safe and effective method for detecting nerve injuries during the placement of TITS screws.

## Figures and Tables

**Figure 1:** (a–i) A 49-year-old man presented with a pelvic fracture (AO/OTA C1.3) due to a fall. (a–c) Preoperative radiographs show bilateral pubic ramus fractures and transforaminal sacral fractures, and the right hemipelvis was vertically displaced. The patient presented with a dysmorphic sacrum. (d) During skeletal traction, the neuroelectrophysiological monitoring alert indicated that the SEP amplitude on the injured side (right) was lower than that on the contralateral side. After reducing the weight of traction, the SEP gradually recovered. (e) Robot-assisted planning for TITS screw fixation. (f, g) Postoperative radiographs showed that the TITS screw was in a good position. (h, i) The fracture healed, and the patient had good functional recovery 16 months postoperatively.

**Table 1:** Summary of the patients.

No.	Age	Sex	Injury mechanism	AO/OTA classification	ISS	Anterior ring injury	Associated injury	Neurological injury (Gibbons' classification)
1	38	M	Fall from height <3 m	C1.3	5	PSS	L 5-7rib fractures; L5 nerve root injury	2
2	47	M	MVA	B2.1	4	Bilateral PRF	None	1
3	19	M	MVA	C2.3	19	Bilateral PRF	L5 S1 nerve root injury; right subtrochanteric femur fracture; L5 transverse process fracture	3
4	60	M	Fall from height >3 m	C3.2	9	Ipsilateral PRF	None	1
5	38	F	Fall from height >3 m	C3.3	13	Bilateral PRF	L3 fracture; TBI; cauda equina syndrome	4
6	39	M	Fall from height >3 m	C1.3	9	Bilateral PRF	None	1
7	35	F	MVA	B2.1	4	Ipsilateral PRF	Right radial head fracture	1
8	42	M	Crush injury	B2.1	9	Contralateral PRF	Chest injury; abdominal injury; S1 nerve root injury	2
9	51	M	Crush injury	C3.2	9	Bilateral PRF+PSS	None	1
10	47	M	Fall from height <3 m	C1.3	4	Ipsilateral PRF	Left tibial fracture	1
11	41	M	Crush injury	C1.3	9	Contralateral PRF	Bilateral calcaneal fracture	1
12	33	M	Fall from height >3 m	C3.3	19	Bilateral PRF	Femoral fracture; sacral plexus nerve injury	3
13	45	F	Fall from height >3 m	C3.3	14	Contralateral PRF	TBI; chest injury; abdominal injury	1
14	61	M	MVA	B2.1	9	Ipsilateral PRF	Tibial plateau fracture	1
15	52	F	PVA	C1.3	19	Ipsilateral PRF	TBI; chest injury; abdominal injury; S1 nerve root injury	2
16	63	M	MVA	C1.3	19	PSS	TBI; spine injury	1
17	49	M	MVA	C1.3	11	Bilateral PRF	Chest injury; abdominal injury; L5 S1 nerve root injury	2
18	23	F	Fall from height >3 m	C3.3	19	Bilateral PRF+ PSS	Bilateral femoral fracture TBI; chest injury; sacral plexus nerve injury	4
19	34	M	MVA	C3.2	13	Bilateral PRF	Chest injury; abdominal injury; spine injury	1
20	52	M	Fall from height >3 m	C3.2	9	Bilateral PRF	Chest injury; spine injury	1
21	34	M	MVA	C1.3	18	Bilateral PRF	Chest injury; abdominal injury; spine injury; L5 S1 nerve root injury	2
22	50	M	MVA	C1.3	4	Bilateral PRF	Abdominal injury	1
	43.32 ± 11.40				11.28 ± 5.54			

MVA: motor vehicle accident; PVA: pedestrian vehicle accident; TBI: traumatic brain injury; PRF: pubic ramus fracture; PSS: pubic symphysis separation.

**Table 2:** Surgical factors, radiological outcomes, and functional outcomes.

No.	Age	Sex	Fixation of anterior ring	Fixation of posterior ring	EBL (ml)	Operation time (min)	TITS (mins)	Fluoroscopy frequency/TITS	FU (mo)	Radiographic grades (Tornetta and Matta)	Functional outcomes (Majeed scores)	Functional outcomes (Majeed score grading)	Neurological injury (Gibbons' classification)
1	38	M	Plate	TITS2	300	120	25	26	12	Excellent	95	Excellent	1
2	47	M	Exfix	TITS2	100	230	20	32	14	Good	98	Excellent	1
3	19	M	Plate	TITS2	900	420	25	28	13	Poor	84	Good	1
4	60	M	CS	TITS1	50	210	25	34	12	Fair	82	Good	1
5^∗^	38	F	Exfix	TITS2	50	120	20	28	18	Good	67	Fair	2
6	39	M	Plate	TITS2	500	165	20	27	12	Excellent	96	Excellent	1
7	35	F	Exfix	TITS1	50	95	40	30	14	Fair	52	Poor	1
8	42	M	CS	TITS2	80	145	35	28	20	Good	80	Good	1
9	51	M	Plate	TITS2	300	435	20	40	13	Excellent	96	Excellent	1
10	47	M	Plate	TITS2	350	210	30	33	14	Excellent	92	Excellent	1
11	41	M	Plate	TITS1	600	150	20	23	18	Excellent	89	Excellent	1
12^∗^	33	M	CS	TITS2	80	245	30	44	12	Good	50	Poor	3
13^#^	45	F	CS	TITS2	50	280	40	32	12	Good	82	Good	1
14	61	M	CS	TITS2	50	265	30	27	16	Excellent	81	Good	1
15	52	F	Plate	TITS2	300	150	30	39	12	Good	80	Good	1
16	63	M	Plate	TITS1	200	120	25	28	14	Good	84	Good	1
17^∗^	49	M	Plate	TITS2	500	180	30	41	16	Good	85	Good	1
18^∗^	23	F	Plate	TITS2	800	180	40	30	12	Good	52	Poor	4
19	34	M	Plate	TITS2	500	200	25	25	14	Excellent	94	Excellent	1
20	52	M	Plate	TITS2	400	130	20	27	18	Excellent	92	Excellent	1
21	34	M	Exfix	TITS1	100	120	35	28	17	Excellent	94	Excellent	1
22	50	M	Plate	TITS2	300	150	30	32	15	Excellent	83	Good	1
	43.32 ± 11.40				298.18 ± 251.82	196.36 ± 90.28	27.95 ± 6.84	31.00 ± 5.56	14.46 ± 2.46		82.18 ± 14.52		

CS: cannulated screw; exfix: external fixator; EBL: estimated blood loss; min: minutes; TITS: transiliac–transsacral screw; FU: follow-up.  ^∗^During the operation, the SEP amplitude on the injured side was lower than that on the contralateral side. ^#^The patient had a spontaneous burst of EMG activity when the guidewire was inserted.

**Table 3:** Comparison study of neurological injury.

Neurological injury	Preoperation	Final follow-up	*P*
Gibbons' classification			0.023^&^
1	13	19	
2	5	1	
3	2	1	
4	2	1	

&: Wilcoxon signed-rank test: *Z* = -2.46, *P* =0.014.

## Data Availability

This article only includes summarized data from this study. Datasets are available from the corresponding author on reasonable request.
